# Identification and functional characterization of mutations in *LPL* gene causing severe hypertriglyceridaemia and acute pancreatitis

**DOI:** 10.1111/jcmm.14768

**Published:** 2020-01-04

**Authors:** Peng Han, Guohong Wei, Ke Cai, Xi Xiang, Wang Ping Deng, Yan Bing Li, Shan Kuang, Zhanying Dong, Tianyu Zheng, Yonglun Luo, Junnian Liu, Yuanning Guan, Chen Li, Subrata Kumar Dey, Zhihong Liao, Santasree Banerjee

**Affiliations:** ^1^ BGI‐Qingdao BGI‐Shenzhen Qingdao China; ^2^ China National GeneBank BGI‐Shenzhen Shenzhen China; ^3^ Department of Endocrinology The First Affiliated Hospital of Sun Yat‐sen University Guangzhou China; ^4^ BGI‐Shenzhen Shenzhen China; ^5^ BGI Education Center University of Chinese Academy of Sciences Shenzhen China; ^6^ Department of Biomedicine Aarhus University Aarhus Denmark; ^7^ Institute of Genetics and Department of Genetics Zhejiang University School of Medicine Hangzhou China; ^8^ Department of Biotechnology Centre for Genetic Studies School of Biotechnology and Biological Sciences Maulana Abul Kalam Azad University of Technology (Formerly West Bengal University of Technology) Kolkata India; ^9^ Brainware university Barasat West Bengal India

**Keywords:** acute pancreatitis, compound heterozygous, hypertriglyceridaemia, *LPL* gene, novel mutations

## Abstract

Hypertriglyceridaemia is a very rare disorder caused by the mutations of *LPL* gene, with an autosomal recessive mode of inheritance. Here, we identified two unrelated Chinese patients manifested with severe hypertriglyceridaemia and acute pancreatitis. The clinical symptoms of proband 1 are more severe than proband 2. Whole exome sequencing and Sanger sequencing were performed. Functional analysis of the identified mutations has been done. Whole exome sequencing identified two pairs of variants in *LPL* gene in the proband 1 (c.162C>A and c.1322+1G>A) and proband 2 (c.835C>G and c.1322+1G>A). The substitution (c.162C>A) leads to the formation of a truncated (p.Cys54*) LPL protein. The substitution (c.835C>G) leads to the replacement of leucine to valine (p.Leu279Val). The splice donor site mutation (c.1322+1G>A) leads to the formation of alternative transcripts with the loss of 134 bp in exon 8 of the *LPL* gene. The proband 1 and his younger son also harbouring a heterozygous variant (c.553G>T; p.Gly185Cys) in *APOA5* gene. The relative expression level of the mutated LPL mRNA (c.162C>A, c.835C>G and c.1322+1G>A) showed significant differences compared to wild‐type LPL mRNA, suggesting that all these three mutations affect the transcription of LPL mRNA. These three mutations (c.162C>A, c.835C>G and c.1322+1G>A) showed noticeably decreased LPL activity in cell culture medium but not in cell lysates. Here, we identified three mutations in *LPL* gene which causes severe hypertriglyceridaemia with acute pancreatitis in Chinese patients. We also described the significance of whole exome sequencing for identifying the candidate gene and disease‐causing mutation in patients with severe hypertriglyceridaemia and acute pancreatitis.

## 1 INTRODUCTION

Hypertriglyceridaemia (HTG) is a very rare autosomal recessive disorder which unlikely causes acute pancreatitis (AP).^1^, ^2^ It has been reported that HTG leads to AP only in 10% of all the cases. Patients with triglyceride (TG) level >2000 mg/dL (22.6 mmol/L) are clinically diagnosed as ‘very severe HTG’, because this level of TG inevitably leads to pancreatitis.^1^, ^3^, ^4^ In addition, patients with fasting TG level in between 1000 (11.3 mmol/L) and 2000 mg/dL (22.6 mmol/L) are diagnosed as ‘severe HTG’, carrying increased risk of developing pancreatitis as TG level may rise above 2000 mg/dL (22.6 mmol/L) after eating. Severe HTG patients with serum TG level >11.3 mmol/L (1000 mg/dL) gradually and progressively developed hepatosplenomegaly, stomach ache, lipaemia retinalis and eruptive xanthomas with an increased risk of AP.^5^, ^6^, ^7^ However, the specific mechanism by which HTG patients gradually develop AP is still unknown. One obvious explanation is that both HTG and increased level of chylomicrons (CM) lead to increase the plasma viscosity, which leads to ischaemia in pancreatic tissue and organ inflammation.^7^, ^8^ Germline mutations in *LPL* gene cause an extremely rare autosomal recessive familial lipoprotein lipase deficiency (LPLD) manifested with severe HTG and chylomicronaemia with recurrent AP.^8^, ^9^ According to the aetiology, HTG is classified into two types, primary and secondary.^9^ In addition, primary HTG is usually caused by germline mutations of lipoprotein lipase (*LPL*) gene. In non‐hepatic tissues, LPL catalyses TG.^3^

The *LPL* gene is located on chromosome 8 and comprises of 10 exons. *LPL* gene encodes an enzyme called lipoprotein lipase, consisting of 475 amino acids.^10^, ^11^ Wild‐type lipoprotein lipase hydrolyses TG in TG‐rich lipoproteins. Homozygous or compound heterozygous mutations in *LPL* gene lead to the complete or partial loss of function of both copies of the *LPL* gene which finally results into severe HTG.^12^ Till date, hundred mutations of *LPL* gene have been reported.^13^

In this study, we identified two unrelated Chinese probands, presented with HTG and AP. Clinical diagnosis found phenotypic heterogeneity between these two probands. The proband 1 was presented with very severe HTG and AP, while the proband 2 was manifested with severe HTG and AP. The clinical phenotype of proband 1 is comparatively more severe than patient 2. Whole exome sequencing identified a novel splice donor site mutation as well as two previously reported mutations in *LPL* gene in these two probands. In vitro functional analysis of these mutations was performed to understand their effect underlying the disease phenotype as well as the phenotypic heterogeneity between these two unrelated Chinese probands. Our present study also strongly described the significance of whole exome sequencing for identifying the candidate gene and disease‐causing mutations in patients with heterogeneous inherited disorders.

## 2 METHODS

### 2.1 Patient and clinical samples

In our present study, we investigated two Chinese probands manifested with HTG and AP, from two unrelated Chinese families. The proband 1 and proband 2 belong to the families 1 and 2, respectively. Moreover, the proband 1 and proband 2 are the only affected individuals in their family. In family 1, we screened the proband 1 (II‐2), proband's mother (I‐2), elder sister (II‐1), wife (II‐2) and his two sons (III‐1 and III‐2). But in family 2, we only screen the proband due to unavailability of blood samples of the other family members. All of the members of these two families have provided informed consent for their participation in this study. The study was approved by the institutional review board at The Ethics Committee of the First Affiliated Hospital, Sun Yat‐sen University.

### 2.2 Whole exome sequencing

Blood samples were collected, and genomic DNA was extracted from these two probands by using a QIAamp DNA Blood Mini Kit (Qiagen) based on the manufacturer's instructions. Both the proband 1 and proband 2 were subjected to whole exome sequencing. Agilent SureSelect version 6 (Agilent Technologies) was used for capturing sequences. Then, the enriched library was sequenced on an Illumina HiSeq 4000. Next, whole exome sequencing reads were aligned to the GRCh37.p.10 by using Burrows‐Wheeler Aligner software (version 0.59). After that, GATK IndelRealigner was used for local realignment of the Burrows‐Wheeler aligned reads. Then, the base quality recalibration of the Burrows‐Wheeler aligned reads was performed by using GATK Base Recalibrator. Next, identification of single‐nucleotide variants (SNV) and insertions or deletions (indel) has been done by GATK Unified Genotyper. After that, annotation of variants has been done with the Consensus Coding Sequences Database (20130630) at the National Center for Biotechnology Information. Illumina pipeline was used for image analysis and base calling. Indexed primers were used for data fidelity surveillance. In order to align the clean sequencing reads with human reference genome (hg19), SOAP aligner (soap2.21) software was used. Then, to assemble the consensus sequence and call genotypes in target regions, we used SOAPsnp (v1.05) software.

Identified variants by whole exome sequencing were selected for data interpretation with minor allele frequency <0.01 in dbSNP, HapMap, 1000 Genomes Project and our in‐house database for 50 000 Chinese Han samples. Based on the variant interpretation guidelines of American College of Medical Genetics and Genomics (ACMG), data interpretation was performed.^14^ Deleterious variations were selected and performed their segregation analysis. The function of the variant and their correlation with the disease phenotype was done by OMIM database and previously published literature. Schematic presentation of the detailed and comprehensive data interpretation process is described in Figure 1.

**Figure 1:** Data interpretation pipeline for whole exome sequencing

### 2.3 Sanger sequencing

Sanger sequencing was performed to validate the variants identified by whole exome sequencing. Sanger sequencing was performed with these primers:

F1 5′‐GGCGCGGGGGTCTCGCGGCG‐3′, R1 5′‐GGCGGCGAATTCTATAGCG‐3′; F2 5′‐GCGCGGTTATATGTCGCGCG‐3′, R2 5′‐GGGCGCATGGTATGCGCGG‐3′; F3 5′‐GGCAGCGTGATTTACGGGC‐3′, R3 5′‐GGCGTATAAGGAGTATACGG‐3′.

The reference sequence NM_000237 of *LPL* was used.

F3 5′‐GCGGATTAGCTGGCCGCGG‐3′, R3 5′‐GCGCTTATAGGCGGTCCGCG‐3′; the reference sequence NM_001166598 of *APOA5* was used.

### 2.4 Exon trapping

#### 2.4.1 Minigene construction

In vitro exon trapping study was performed to understand the effect of the splice donor site mutation (c.1322+1G>A) of the *LPL* gene at the transcriptional level. Minigene construction has been done according to the previously reported protocol.^15^ The genomic DNA from proband 1 and proband 2 was used as template for constructing minigene. Minigenes were consisting of one wild‐type (WT) and one mutant allele, including exon 7, intron 7, exon 8, intron 8 and exon 9 with 5′ and 3′ intronic flanking sequences. Minigenes were amplified by PCR and cloned into pSPL3 (exon trapping vector) vector through double digestion by two restriction endonucleases: *BamHI* and *XhoI*.^15^ After constructing both the wild‐type and mutant minigenes, they were transiently transfected into COS‐7 cell line.

#### 2.4.2 Transfection and Sanger sequencing

Dulbecco's modified Eagle's medium supplemented with 10% foetal bovine serum, 1% penicillin‐streptomycin and 1% glutamine was used to culture the COS‐7 cells within a humidified incubator with 5% CO_2_ and 37°C temperature. Total RNA was extracted with TRIzol (Takara Biomedical Technology (Beijing) Co., Ltd.) after 48 hours of transfection. Then, 5 μg of RNA in a total volume of 20 μL with SuperScript II RNAse H‐Reverse Transcriptase and oligo‐dT priming (Takara Biomedical Technology (Beijing) Co., Ltd.) was used to prepare cDNA. After that, cDNA was amplified by the vector primers SD6 (5′‐TCTGAGTCACCTGGACAACC‐3′) and SA2 (5′‐ATCTCAGTGGTATTTGTGAGC‐3′), according to the recommended PCR reaction condition. Lastly, the amplified products were separated on a 2% TBE agarose gel and subjected to Sanger sequencing.

### 2.5 Construction of wild‐type and mutant human LPL recombination plasmid

pEGFP‐N1‐LPL‐WT vector (Shanghai Sunny Biotechnology Co., Ltd.) containing normal human LPL cDNA was used as template to generate site‐directed mutagenesis. These three (c.162C>A, c.835C>G and c.1322+1G>A) mutations were introduced into LPL cDNA by mutagenic primers:

The primer pairs used for site‐directed mutagenesis of these three mutations (c.162C>A, c.835C>G and c.1322+1G>A) are listed as follows:

pEGFP‐N1‐LPL‐M162‐F′5′‐AGGACACTTGACACCTCATTC‐3′, pEGFP‐N1‐LPL‐M162‐R′ 5′‐GAATGAGGTGTCAAGTGTCCT‐3′; pEGFP‐N1‐LPL‐M835‐F′5′‐CATCGACTCTGTGTTGAATGAAG‐3′, pEGFP‐N1‐LPL‐M835‐R′5′‐CTTCATTCAACACAGAGTCGATG‐3′; pEGFP‐N1‐LPL‐M1322‐F′5′‐GCGAAGATATCTCATCCATG‐3′; pEGFP‐N1‐LPL‐M1322‐R′ 5′‐GGCTGCCTGCGGTGGAGTGCG‐3′; and pEGFP‐N1‐LPL‐F′5′‐GTCACTCGAGGCTAGCATGGAGAGCAAAGC‐3′ contain *XhoI* site, and pEGFP‐N1‐LPL‐R′5′‐GTCACTGCAGACCGGTGCGCCTGACTTCA‐3′ contains *Pst1* recognition site.

Primers of pEGFP‐N1‐LPL‐F and pEGFP‐N1‐LPL‐R contain *XhoI* and *PstI* recognition sites, which were used to amplify mutant plasmid M162‐pEGFP, M835‐pEGFP and M1322‐pEGFP. The final PCR amplification was inserted into the digested pEGFP‐N1. Recombined plasmids were transformed into *Escherichia coli* DH5α. DNA was prepared by NucleoBond Xtra Midi Kit (MN). Sequence was verified by Sanger sequencing.

### 2.6 COS‐7 cell transfection

COS‐7 cell maintained in Dulbecco's modified Eagle's medium (DMEM, HyClone) supplemented with 10% foetal bovine serum (HyClone) at 37°C in a 5% CO_2_ environment (HF240 CO_2_ incubator, Heal Force). COS‐7 cells were plated at 3 × 10^4^ per well into six‐well plates and cultured overnight. The WT, mutant and empty control vector were transient transfected into COS‐7 cells using PolyJet (SignaGen Laboratories). After culturing for 24 hours, heparin sodium was added (the final concentration was 200 mU/mL) and the culture lasted for 12 hours. The supernatant and cells were collected, respectively.

### 2.7 Real‐time PCR (RT‐PCR)

Transfected COS‐7 cells were collected, and total RNA was extracted using TRIzol Reagent (Takara Biomedical Technology (Beijing) Co., Ltd.). Reverse transcription was then performed using PrimeScript™ RT Reagent Kit (Takara Biomedical Technology (Beijing) Co., Ltd.). The amplification conditions for *LPL* gene and 18S rRNA were as follows: initial denaturation at 95°C for 10 seconds, amplification phase (denaturation at 95°C for 5 seconds, annealing at 60°C for 30 seconds and extension at 70°C for 15 seconds) performed for 40 cycles, dissolution curve period at 60°C for 1 minutes and finally 95°C for 15 seconds.

RT‐PCR was performed by ABI 7500 real‐time PCR system (Applied Biosystems). The relative expression level was calculated using 2^−ΔΔCt^, and the software SPSS20 was used for the analysis of the data.

The relative expression level of *LPL* gene was evaluated by real‐time PCR by using these primer sequences, which are as follows: LPL 5′‐AAGAACCGCTGCAACAATCT‐3′, 5′‐GGCAGAGTGAATGGGATGTT‐3′.

18SrRNA (internal reference) 5′‐cctggataccgcagctagga‐3′, 5′‐gcggcgcaatacgaatgcccc‐3′.

### 2.8 Analysis of LPL activity and mass

Post‐heparin transfected COS‐7 cell culture medium was harvested and centrifuged at 4°C for 20 minutes at  12 000 *g*. The remaining precipitated cells were washed with PBS and then solubilized in 80 μL cell lysis buffer (Tiangen Biotechnology Co., Ltd.). The cell lysates were centrifuged at 4°C for 20 minutes at 12 000 *g*, and the supernatant was stored at −80°C. LPL mass and activity were determined by Human LPL ELISA kit (Shanghai Xinfan Biotechnology Co., Ltd.) and LPL activity assay kit (Cell Biolabs, INC.), respectively, by using M5 full‐band multifunctional enzyme label instrument (Molecular Devices). In addition, for LPL activity assay, the parameters were set to 485/520 nm and filter set with cut‐off of 495 nm.

### 2.9 Evolutionary conservation test

To understand the evolutionary conservation of the wild‐type amino acids of the missense mutation (c.835C>G; p.Leu279Val) in *LPL* gene, sequence alignment between human (*Homo sapiens*) (GenBank Accession: NM_000237.3), bovine (*Bos taurus*) (GenBank Accession: NM_001075120.1), sheep (*Ovis aries*) (GenBank Accession: NM_001009394.1), chicken (*Gallus gallus*) (GenBank Accession: NM_205282.1), rat (*Rattus norvegicus*) (GenBank Accession: NM_012598.2) and mouse (*Mus musculus*) (GenBank Accession: NM_008509.2) was performed.

## 3 RESULT

### 3.1 Pedigree and family

In this present study, we identified two Chinese patients from two unrelated Chinese families, manifested with severe HTG and AP (Figure 2A,B). In both the families, only the proband is the affected individual. We clinically diagnosed the proband 1 with very severe HTG and AP, while the proband 2 was identified with severe but comparatively milder phonotype than proband 1. Here, we aimed to identify the candidate gene and disease‐causing mutation underlying the disease phenotype in both of these two probands and functionally characterize the variants by performing in vitro experiments. In vitro functional analysis allowed us to understand the basis of phenotypic heterogeneity between these two patients. In addition, proband 1 and all the living members of his family have been studied well, whereas proband 2 is the only member of her family has been studied due to the early death of her parents. The lipid profiles of all the subjects are described in Table 1. Routine blood test result of all the subjects is given in Table 2.

**Figure 2:** A‐B, Family pedigree of proband 1 (A) and proband 2 (B). The filled symbol indicates the patient (proband), and the half‐filled symbol indicates the unaffected and heterozygous carrier parents. The arrow points to the proband. C‐F, Computed tomography (CT) test. (C) Arterial phase of CT enhanced scan. The white arrow indicates the disappearance of fat gap between pancreas and stomach, and local effusion. The black arrow indicates the slight oedema at both the body and tail of the pancreas. (D) Coronal reconstruction of CT enhanced scan. The white arrows indicate the peripancreatic exudation. (E) Arterial phase of CT enhanced scan. The white arrows indicate exudation and effusion beneath the body of the pancreas. (F) Sagittal reconstruction of CT enhanced scan. The white arrows indicate peripancreatic exudation

**Table 1:** The lipid profiles of all the subjects

Lipids	Reference range	Proband 1 (II‐2)	Mother of proband 1 (I‐2)	Sister of proband 1 (II‐1)	Wife of proband 1 (II‐3)	Elder son of proband 1 (III‐1)	Younger son of proband 1 (III‐2)	Proband 2 (II‐1)
Triglyceride	0.33‐1.70 (mmol/L)	21.51↑	1.46	0.65	0.49	0.77	0.81	3.8↑
Total cholesterol	3.10‐5.70 (mmol/L)	5.6	5.15	4.18	3.6	3.31	4.13	2.85↓
Low‐density lipoprotein cholesterol	1.94‐3.61 (mmol/L)	1.52↓	3.43	2.52	2.1	2.06	2.66	1.61↓
High‐density lipoprotein cholesterol	1.09‐1.63 (mmol/L)	0.33	1.04	1.22	1.35	0.85↓	1.06	0.68↓
Apolipoprotein E	27.0‐45.0 (mg/L)	60↑	39.9	37.6	38	29.4	35.4	63.2↑
Apolipoprotein A1	0.60‐2.00 (g/L)	0.78	1.26	1.26	1.29	1.02	1.07	1.14
Apolipoprotein B	0.35‐1.75 (g/L)	0.42	1.1	0.69	0.58	0.6	0.76	0.53
Lipoprotein (a)	60‐300 (mg/L)	25↓	35	56	88	118	131	48
Fat turbidity index	0.00‐0.10	4↑	0	0	0	0	0	0
The condition when blood taken		Fenofibrate 200 mg QD and AP attack						Fenofibrate 200 mg QD and strict dietary restriction

**Table 2:** Routine blood test result of all the subjects

Blood examination results	Reference range	Proband 1 (II‐2)	Mother of proband 1 (I‐2)	Sister of proband 1 (II‐1)	Wife of proband 1 (II‐3)	Elder son of proband 1 (III‐1)	Younger son of proband 1 (III‐2)	Proband 2 (II‐1)
Albumin	35.0‐50.0 (g/L)	50.7↑	43	41.4	47.5	42.4	45.8	45.8
Prealbumin	200‐400 (mg/L)	2↓	282	225	261	181↓	202	271
Total protein	64.0‐87.0 (g/L)	76	73	73	78	68	70	75
Alkaline phosphatase	30‐120 (U/L)	71	82	75	69	264↑	312↑	56
Alanine aminotransferase	1‐40 (U/L)	29	31	24	22	16	23	14
Aspartate aminotransferase	1‐37 (U/L)	57↑	30	28	24	40↑	47↑	21
Cholinesterase	5300‐12 900 (U/L)	7855	8690	9676	5943	8690	8507	7831
γ‐Glutamic transpeptidase	2‐50 (U/L)	10	30	16	18	11	11	12
Leucine aminopeptidase	30‐70 (U/L)	46	52	62	56	69	69	38
Lactate dehydrogenase	114‐240 (U/L)	298↑	249↑	240	190	327↑	314↑	209
Glutamate dehydrogenase	0.1‐7.5 (U/L)	8.4↑	17.8↑	2.7	2.5	1.6	2.6	1.5
Total bilirubin	3.0‐22.0 (umol/L)	12.3	7.4	5.7	16.7	7	8.9	9.2
Direct bilirubin	0.5‐7.0 (μmol/L)	1.8	1	1.1	3.3	1.4	1.4	1.8
Bile acid	0.1‐10.0 (μmol/L)	2.5	2.4	1.2	2.5	3.3	1.4	7.4
Glucose	2.9‐6.0 (mmol/L)	3	3.9	3.6	3.6	3.2	3.2	5.5
Uric acid	Female: 140‐360; Male: 140‐430 (μmol/L)	329	369↑	298	213	291	290	194
Creatinine	53‐115 (μmol/L)	90	78	47↓	43↓	34↓	29↓	60
Urea	2.9‐8.6 (mmol/L)	5.6	5.9	4.9	3	4	5.8	4.2
Potassium (mmol/L)	3.5‐5.3 (mmol/L)	3.7	3.8	3.7	3.9	3.8	4.4	4
Sodium (mmol/L)	135‐145 (mmol/L)	138	143	140	140	142	141	140
Chlorine (mmol/L)	96‐110 (mmol/L)	103	107	106	105	107	106	104
Calcium (mmol/L)	2.10‐2.60 (mmol/L)	2.44	2.27	2.35	2.36	2.42	2.46	2.42
Phosphorus (mmol/L)	0.97‐1.62 (mmol/L)	0.94↓	1.18	1.46	1.02	1.63↑	1.75↑	1.24
Carbon dioxide (mmol/L)	20‐30 (mmol/L)	23	23	20	22	22	20	24
Total cholesterol (mmol/L)	3.10‐5.70 (mmol/L)	4.78	5.15	4.18	3.6	3.31	4.13	2.85↓
Low‐density lipoprotein cholesterol (mmol/L)	1.94‐3.61 (mmol/L)	1.83↓	3.43	2.52	2.1	2.06	2.66	1.61↓
High‐density lipoprotein cholesterol (mmol/L)	1.09‐1.63 (mmol/L)	0.24↓	1.04↓	1.22	1.35	0.85↓	1.06↓	0.68↓
Triglyceride (mmol/L)	0.33‐1.70 (mmol/L)	12.18↑	1.46	0.65	0.49	0.77	0.81	3.8↑
Apolipoprotein E	27.0‐45.0 (mg/L)	68↑	39.9	37.6	38	29.4	35.4	63.2↑
Apolipoprotein A1	0.60‐2.00 (g/L)	0.55↓	1.26	1.26	1.29	1.02	1.07	1.14
Apolipoprotein B	0.35‐1.75 (g/L)	0.12↓	1.1	0.69	0.58	0.6	0.76	0.53
Lipoprotein (a)	60‐300 (mg/L)	25↓	35↓	56↓	88	118	131	48↓
Fat turbidity index	0.00‐0.10	4↑	0	0	0	0	0	0
Haemolytic index	0.00‐010	2↑	0	0	0	0	0	0
Icteric index	0.00‐0.10	0	0	0	0	0	0	0
The condition when blood taken		Fenofibrate 200 mg QD + Acipimox 250 mg TID + Fish oil						Fenofibrate 200 mg QD and strict dietary restriction

### 3.2 Clinical description

#### 3.2.1 Patient 1

The proband 1 is a 32‐year‐old Chinese man belongs to nonconsanguineous Chinese parents (Figure 2A). At the age of 25 years, the proband was first identified with severe HTG when he was admitted in our hospital with severe AP. Since then, he experienced stomach ache due to AP, once in every 2‐3 months in the first 5 years after clinical diagnosis but gradually the frequency of the AP‐induced stomach ache reduced (once in every 4‐12 months without obvious inducing factor). However, sometimes mild stress also triggered his stomach ache due to AP. Interestingly, in the proband, we identified that the serum TG was 30 mmol/L at the time of stomach ache due to AP but the serum TG level was decreased to 10‐20 mmol/L when the patient experienced no AP‐induced stomach ache. After the patient was experienced with AP at first time, we recommended him and start fenofibrate treatment. Gradually, AP was resolved by octreotide and omeprazole treatment accompanied with restricted diet. In 2016, he once experienced a severe liver damage and rhabdomyolysis due to the combination therapy of atorvastatin and fenofibrate. Presently, he is under the treatment of fenofibrate 200 mg QD, acipimox 250 mg TID and fish oil 1‐2 capsules, with strict and restricted diet.

The proband had never been identified with hypertension, diabetes, coronary heart disease or any other diseases. His parents were born and brought‐up at the same town but not consanguineous. His father had been suffering from hepatitis and accidentally died at age of 57. The blood lipids' levels for his mother, sister and two sons were all normal (Table 1). The full blood test result is given in Table 2.

Abdominal computed tomography (CT) showed pancreatic oedema, both at the pancreatic body and at the tail. No haemorrhage or necrosis was identified in pancreas. Enhanced scan showed uniform enhancement of the pancreas, blurred fat space and a small amount liquid density shadow around the pancreas. The pancreas head was not enlarged, and the pancreatic duct was not dilated, AP was clinically diagnosed. Other abnormities have been identified which includes the calcification at S5 of liver, muddy stones inside the gall bladder and common bile duct, splenomegaly and multiple small cysts at both the kidneys (Figure 2C‐F).

#### 3.2.2 Patient 2

The proband 2 is a 42‐year‐old Chinese woman presented with HTG and AP (Figure 2B). The proband 2 was first admitted at our hospital at the age of 36 years with AP. She was also identified with HTG (TG: 17.1 mmol/L). We recommend her with the treatment of fenofibrate 200 mg QD. After treatment, the TG levels was controlled (TG: 5.1‐10.2 mmol/L) with no recurrence of AP. Including the present medication and strict dietary restriction, her TG level was reduced to 3.8 mmol/L.

In summary, according to the clinical data, comparing with proband 2, proband 1 showed more severe HTG with increased apolipoprotein E, accompanied by frequent occurrence of AP. In proband 2, the treatment outcome is fair well with fenofibrate 200 mg QD and strict dietary restriction. Atorvastatin, combined with fenofibrate, induced the severe side‐effect of liver damage and rhabdomyolysis for the proband 1.

### 3.3 Identification of a novel splice donor site mutation in the *LPL* gene

#### 3.3.1 Proband 1

In the proband 1, whole exome sequencing identified two heterozygous mutations (c.162C>A and c.1322+1G>A) in the *LPL* gene and a heterozygous mutation (c.553G>T) in *APOA5* gene (Figure 3A). The heterozygous transversion, c.162C>A in exon 2, leads to the formation of a premature stop codon followed by the formation of a truncated (p.Cys54*) LPL protein of 53 amino acids compared with the wild‐type LPL protein of 475 amino acids. Hence, it is a *loss‐of‐function* mutation. The heterozygous splice donor site mutation, c.1322+1G>A in the first nucleotide of intron 8, leads to the loss of wild‐type donor splice site followed by the aberrant splicing of LPL mRNA which finally results in the formation of alternative transcripts. The heterozygous missense mutation (c.553G>T) in *APOA5* gene leads to the replacement of glycine by cysteine (p.Gly185Cys). Sanger sequencing revealed that the proband inherited the splice donor site (c.1322+1G>A) mutation from his mother, while the nonsense (c.162C>A) mutation is a de novo mutation (Figure 3A). Proband's elder sister (II‐1) did not carry any of these three heterozygous mutations. Proband's elder son (III‐1) was harbouring the heterozygous nonsense (c.162C>A) mutation, whereas proband's younger son (III‐2) was carrying the splice donor site mutation (c.1322+1G>A) and the missense mutation (c.553G>T; Figure 3A). According to the variant interpretation guidelines of American College of Medical Genetics and Genomics (ACMG), these two variants (c.162C>A and c.1322+1G>A) were classified as *“likely pathogenic”* variants.

**Figure 3:** Sanger Sequencing. Partial DNA sequences in the *LPL* gene and *APOA5* gene by Sanger sequencing of the proband 1 and his family members (A). Partial DNA sequences in the *LPL* gene by Sanger sequencing of the proband 2 (B). The reference sequence NM_000237 of *LPL* gene was used. The reference sequence NM_001166598 of *APOA5* gene was used

These two mutations (c.162C>A and c.1322+1G>A) in *LPL* gene were co‐segregated well with the disease phenotype in the family with an autosomal recessive mode of inheritance. We did not find these two mutations 100 ethnically matched normal healthy control individuals. These two mutations were also not present in the ExAC, dbSNP, gnomAD, 1000 Genome Database as well as in BGI's database which is consisting of ~50 000 Chinese Han samples. Hence, both of these two mutations could be regarded as potential pathogenic mutations, causes disease in proband 1 in a compound heterozygous manner.

#### 3.3.2 Proband 2

In the proband 2, whole exome sequencing identified two heterozygous mutations (c.835C>G and c.1322+1G>A) in the *LPL* gene (Figure 3B). The heterozygous transversion, c.835C>G in exon 6, leads to the replacement of a leucine by valine at the position of 279 amino acid (p.Leu279Val) of the wild‐type LPL protein. The heterozygous splice donor site mutation, c.1322+1G>A in the first base of intron 8, leads to the loss of wild‐type donor splice site followed by the formation of alternative transcripts. As proband's parents were already died, we were unable to test them for these two heterozygous mutations.

These two mutations were not detected in 100 ethnically matched normal healthy control individuals. These two mutations were also not present in the ExAC, dbSNP, gnomAD, 1000 Genome Database as well as in BGI's database which is consisting of ~50 000 Chinese Han samples. Hence, both of these two mutations could be regarded as potential pathogenic mutations, causes disease in proband 2 with compound heterozygosity.

### 3.4 Functional analysis of the novel splice donor site mutation

In vitro exon trapping assay found that the novel heterozygous splice donor site (c.1322+1G>A) mutation at the first nucleotide of intron 8 of the *LPL* gene disrupts the wild‐type LPL exon 8 splice donor site. Partial genomic DNA constructs consisting of exons 7, 8 and 9 of *LPL*, with or without the splice site mutation, were expressed in COS‐7 cells. Reverse transcription‐PCR and direct sequencing of LPL cDNA from cells transfected with the wild‐type construct showed normal splicing of exon 7 to exon 9. In contrast, direct sequencing of mutant reverse transcription‐PCR products revealed partial loss of 134 bp from exon 8 which in turn results in removal or loss of 45 amino acids in the LPL polypeptide due to complete abolition of the wild‐type donor splice site (Figure 4A‐C).

**Figure 4:** Functional characterization of the splice donor site mutation by in vitro exon trapping assay. (A) RT‐PCR products of the c.1322+1G>A in pSPL3 minigene constructs, Lane M: the 1000 bp marker/ladder. Lanes 1 and 2: the wild‐type (WT) correctly spliced exon 7, exon 8 and exon 9 of LPL cDNA in proband 1 and proband 2, respectively. Lanes 3 and 4: the aberrantly spliced LPL cDNA with skipping of 134 bp of exon 8. Lanes 5 and 6: empty vector 265 bp. Lanes 7 and 8: the negative control. (B) Schematic representation of the splicing model. (C) Reverse transcription‐PCR and direct sequencing of LPL cDNA from cells transfected with the wild‐type construct showed normal splicing of exon 7 to exon 9. In contrast, Sanger sequencing of mutant reverse transcription‐PCR (RT‐PCR) products revealed partial loss of 134 bp from exon 8 which in turn results in removal of 45 amino acids in the LPL polypeptide due to abolition of the wild‐type donor splice site

### 3.5 In vitro functional analysis of *LPL* mutants

#### 3.5.1 Relative expression of mRNA

LPL mRNA has been extracted from transfected COS‐7 cells and analysed by fluorescent RT‐PCR. The result showed that the relative expression of LPL mRNA with any of these three mutations (c.162C>A, c.835C>G and c.1322+1G>A) was significantly lower compared to wild‐type LPL mRNA, suggesting that these three mutations affect the transcription of *LPL* gene (Figure 5A). Each experiment was repeated three times.

**Figure 5:** Functional analysis of LPL mutants in vitro*.* (A) Quantitation of extracted mRNA and normalized to 18S rRNA. mRNA was extracted from transfected COS‐7 cells containing the mutant *LPL* genes and quantitatively determined by qPCR. The expression level of LPL mRNA was showing significant difference between the wild‐type and mutants (c.162C>A, c.835C>G and c.1322+1G>A). Values are shown as mean ± SD. (B) Lipase mass analysis of wild‐type and *LPL* mutants in both the cell culture medium and the cell lysates was performed. Lipase mass was measured by ELISA. There was no significant difference found in lipid mass in both cell culture medium and the cell lysate between the wild‐type and mutants. Values are shown as mean ± SD. (C) Lipase enzyme activity analysis of wild‐type and *LPL* mutants in both the cell culture medium and the cell lysates was performed. Lipase enzyme activity of *LPL* mutants was assayed as a percentage of LPL wild‐type after transfection. There was significant difference found in LPL enzyme activity between the wild‐type and mutants in cell culture medium but not in cell lysate. Values are shown as mean ± SD

### 3.6 Analysis of LPL mass and LPL enzyme activity

In order to understand the significance of the c.162C>A, c.835C>G and c.1322+1G>A mutations, constructs containing the above mutations were transformed into the COS‐7 cells. LPL mass and LPL enzyme activity in both cell culture medium and cell lysate were analysed by ELISA and enzyme fluorescent method, respectively. Our result clearly showed that the COS‐7 cells transfected with wild‐type LPL cDNA presented a steady or persistent levels of LPL mass and LPL enzyme activity in both cell culture medium and cell lysate (Figure 5B,C). However, COS‐7 cells separately transfected with all of these three LPL (c.162C>A, c.835C>G and c.1322+1G>A) mutations showed comparatively consistent level of LPL mass in both cell culture medium and cell lysate (Figure 5B). Interestingly, our result also showed significant decrease in LPL enzyme activities in all of these three mutant‐construct transfected COS‐7 cells in cell culture medium (Figure 5C), but there was no significant difference in LPL enzyme activities between wild‐type and mutant‐construct transfected COS‐7 cells in cell lysate (Figure 5C).

### 3.7 Evolutionary conservation test

In the proband 2, whole exome sequencing identified a heterozygous transversion, c.835C>G in exon 6, leads to the replacement of a leucine by valine at the position of 279 amino acid (p.Leu279Val) of the wild‐type LPL protein. Multiple sequence alignment showed that p.Leu279 is evolutionarily highly conserved among different species, indicating its importance in both the structure and the functions of the wild‐type LPL protein (Figure 6A).

**Figure 6:** In silico analysis of LPL mutations. (A) To understand the evolutionary conservation of the wild‐type amino acids of the missense mutation of *LPL* gene to perform sequence alignment between human (*Homo sapiens*) (GenBank Accession: NM_000237.3), bovine (*Bos taurus*) (GenBank Accession: NM_001075120.1), sheep (*Ovis aries*) (GenBank Accession: NM_001009394.1), chicken (*Gallus gallus*) (GenBank Accession: NM_205282.1), rat (*Rattus norvegicus*) (GenBank Accession: NM_012598.2) and mouse (*Mus musculus*) (GenBank Accession: NM_008509.2). The red coloured box showed that amino acid p.Leu279 is evolutionarily highly conserved. (B) Crystal structure of the whole LPL protein (PDB ID: http://www.rcsb.org/pdb/search/structidSearch.do?structureId=6E7K) and predicted LPL protein structure upon these three mutations have been shown separately. (C) The p.Leu279 of the wild‐type LPL protein showed no clash. (D) The mutated residue p.Val279 causes one clash marked with “yellow” line

### 3.8 In silico protein structural analysis

In order to understand the effect of the missense mutation (c.835C>G) on the LPL protein structure, in silico protein structural analysis was performed, based on the LPL crystal structure (PDB ID: http://www.rcsb.org/pdb/search/structidSearch.do?structureId=6E7K) in PDB database (Figure 6B‐E). The wild‐type LPL protein and all of these three mutations (c.162C>A, c.1322+1G>A and c.835C>G) and their effect on LPL protein are shown in Figure 6B. We used Chimera (https://www.cgl.ucsf.edu/chimera/) to analysis the clash occurred after missense mutation. The replacement of leucine by valine (c.835C>G, p.Leu279Val) results into the occurrence one clash. The p.Leu279 is shown in Figure 6C. The mutated residue p.Val279 causes one clash marked with “yellow” line (Figure 6D).

## 4 DISCUSSION

In the present study, we identified two Chinese probands with severe HTG and AP. Proband 1 was presented with very severe HTG and AP, while proband 2 was manifested with similar but relatively less serious HTG phenotype than proband 1. In the proband 1, whole exome sequencing identified two heterozygous mutations (c.162C>A and c.1322+1G>A) in the *LPL* gene. In the proband 2, whole exome sequencing also identified two heterozygous mutations (c.835C>G and c.1322+1G>A) in the *LPL* gene.

The heterozygous transversion, c.162C>A in exon 2, leads to the formation of a premature stop codon followed by the formation of a truncated (p.Cys54*) LPL protein of 53 amino acids compared with the wild‐type LPL protein of 475 amino acids. Therefore, the p.Cys54* mutation downstream is not translated. It is expected that this very short truncated peptide lack off catalytic function. Hence, it is a *loss‐of‐function* mutation. In 2006, Chan et al^16^ reported this mutation (c.162C>A) together with a homozygous mutation (754C>G) in *LPL* gene in a Chinese baby girl with HTG.

In this study, both the probands are carrying the same novel heterozygous splice donor site (c.1322+1G>A) mutation in *LPL* gene. It is a heterozygous transition (G>A) at the first nucleotide of the intron 8 of the *LPL* gene. Hence, it is a splice donor site mutation which is located at canonical splice site. In order to understand the effect of this mutation at transcriptional level, we performed in vitro exon trapping assay. In vitro exon trapping assay found that this novel heterozygous splice donor site (c.1322+1G>A) mutation of the *LPL* gene disrupts the wild‐type LPL exon 8 splice donor site in both the probands and causes partial loss of 134 bp from exon 8 which in turn results in removal or loss of 45 amino acids in the LPL polypeptide due to complete abolition of the wild‐type donor splice site (Figure 4B,C).

However, the heterozygous transversion, (c.835C>G, p.Leu279Val), has been frequently reported and well‐studied. In 2014, Chan et al^17^ reported the first case report with the presence of heterozygous p.Leu279Val in a Chinese patient with HTG and AP. It has been reported that in Asian countries (Thailand, Mainland China, Taiwan and Hong Kong), the frequency of p.Leu279Val varied from 1/160 to 5/101, while it has never been reported in European population.^9^, ^17^, ^18^, ^19^, ^20^, ^21^ Therefore, the genetic variations in *LPL* gene showed extreme heterogeneity among different races and ethnicity. In Asian population, p.Leu279Val is a well‐reported pathogenic mutation leads to LPL deficiency with the founder effect.^3^, ^16^ In addition, both in vitro studies and biomedical methods confirmed the pathogenicity of the p.Leu279Val, while there has been no in vivo research to elucidate its particular pathogenic mechanism.^17^, ^19^ In addition, p.Leu279 may involve in the catalytic function of LPL, as it acts as a heparin‐binding site by constituting two disulphide bridges (p.Cys278‐p.Cys283) and (p.Cys264‐p.Cys275).^18^, ^19^ Multiple‐species sequence alignment results showed that p.Leu279 was evolutionarily highly conserved, which indicates the significance of p.Leu279 in both the structure and function of wild‐type LPL protein.

Here, we also identified a heterozygous missense variant (c.553G>T; p.Gly185Cys) in *APOA5* gene in the proband 1 (II‐2) and his younger son (III‐2). This is a well‐reported variant in Chinese population.^22^, ^23^ In 2003, Kao et al^22^ reported that c.553G>T, in the *APOA5* gene, is associated with HTG. Later, Tang et al^23^ reported that c.553G>T in the *APOA5* gene is associated with an increased risk of developing coronary artery disease and altered TG levels in a Chinese population. Previously, we also presumed that the severe HTG and AP in proband 1 (II‐2) were bigenic and caused by both the mutations of *LPL* gene and the heterozygous mutation of *APOA5* gene. In contrast, Sanger sequencing confirmed that this variant was also present in the younger son (III‐2) of the proband but he is phenotypically normal. So, we exclude this variant as a pathogenic variant in this family though this variant was reported to cause HTG or increased risk of developing coronary artery disease and altered TG levels in Chinese population.

Lipoprotein lipase (LPL) is an important enzyme majorly involved in the metabolism of TG.^24^ In HTG patients, germline mutations in LPL gene cause low levels of plasma LPL activity.^25^, ^26^ Structurally, LPL protein comprises of two domains: a large N‐terminal domain (amino acid residues 1‐315) with catalytic centre and active site region mainly involved in heparin and substrate binding and a small C‐terminal domain (amino acid residues 316‐448) mainly involved in stability and activity of LPL enzyme with the formation of the LPL head‐to‐tail noncovalent homodimer, a configuration essential for the activity of the enzyme.^27^, ^28^ Although HTG with AP is very rare disease phenotype among patients but till now, only 200 disease‐causing mutations were identified. Among these 200 mutations, 70% are missense, 10% are nonsense, 18% are rearrangements, and remaining 2% are unknown mutations.

In this study, our result showed that these three mutations (c.162C>A, c.835C>G and c.1322+1G>A) majorly affect the stability of transcription and significantly decrease the expression of *LPL* gene compared with the wild‐type (Figure 5A). In order to understand the effect of the c.162C>A, c.835C>G and c.1322+1G>A mutations on LPL mass and LPL enzyme activity in both cell culture medium and cell lysate, we performed ELISA and enzyme fluorescent method, respectively. Our result clearly showed that the COS‐7 cells separately transfected with all of these three LPL (c.162C>A, c.835C>G and c.1322+1G>A) mutations showed comparatively consistent level of LPL mass in both cell culture medium and cell lysate (Figure 5B). However, significant decrease in LPL enzyme activities was found in all of these three mutant‐construct transfected COS‐7 cells in cell culture medium (Figure 5C), but no change in cell lysate (Figure 5C). Hence, these three mutations exhibited both decreased catalytic activity and secretion ability.

HTG with AP is an extremely rare disorder of lipoprotein metabolism caused by germline mutations in *LPL* gene with an autosomal recessive mode of inheritance. In this study, we identified a novel and two previously reported mutations in the *LPL* gene causing HTG and AP. HTG with AP is an extremely severe and potentially fatal.^1^, ^3^ However, very severe and severe HTG generally develop with genetic mutations in *LPL* gene which impair the catabolism of TG in CM and very low‐density lipoproteins (VLDL).^10^ In adipose tissue, muscle, islets and macrophages, lipoprotein lipase is playing the key role in hydrolysis of the TG in CM and VLDL.^29^ Hence, mutations in *LPL* gene cause the formation of partially or completely non‐functional lipoprotein lipase which cannot catabolize the TG in CM leads to the gradual and progressive increase in CM levels and increased the risk for AP, HTG, diabetes mellitus and other metabolic disorders.^30^ In order to provide specific and effective treatment to the patients with type I hypertriglyceridaemia, analysis of LPL mass and LPL enzyme activity is very crucial and significant.^31^ Patients with no LPL mass could not be successfully treated with alipogene tiparvovec due to immune response to the injected functional LPL protein.^32^ Hence, analysis of both lipid mass and lipase enzyme activity assay is very significant for the patients with HTG and AP. In our present study, we identified two unrelated Chinese patients from two Chinese families. Both probands were identified and clinically diagnosed with HTG and AP. Proband 1 has been suffering from very severe HTG with AP, while the proband 2 was identified with severe HTG. Whole exome sequencing identified two pairs (c.162C>A and c.1322+1G>A in proband 1 and c.835C>G and c.1322+1G>A in proband 2) of variants in *LPL* gene in both the probands. Both the probands was found to harbour a common splice donor site mutation (c.1322+1G>A). Proband 1 was identified with a nonsense mutation (c.162C>A; p.Cys54*), while proband 2 was carrying a missense mutation (c.835C>G, p.Leu279Val). The effect of a nonsense truncated protein is more than that of a protein with a missense change. Hence, proband 1 was identified with more severe phenotype than proband 2.

In conclusion, in this study, we identified two unrelated Chinese patients with extremely rare and severe HTG with AP. Both the patients sharing a common splice donor site mutation in *LPL* gene. Phenotypic heterogeneity was also identified between these two patients. Functional characterization of identified mutations has been done. Additionally, we also described the importance of whole exome sequencing for identifying candidate gene with disease‐causing mutations in rare disease of metabolism.

## CONFLICT OF INTEREST

The authors confirm that there are no conflicts of interest.

## AUTHOR CONTRIBUTIONS

Santasree Banerjee and Zhihong Liao designed the study and supervised the project. Peng Han, Guohong Wei, Ke Cai and Xi Xiang conducted acquisition and analysis of all the clinical data. Wang Ping Deng, Yan Bing Li, Han Peng, Junnian Liu and Yuanning Guan made WES pipeline. Shan Kuang, Tianyu Zheng, Zhanying Dong and Yuanning Guan analysed the data. Santasree Banerjee, Shan Kuang and Peng Han wrote the manuscript. Santasree Banerjee, Zhihong Liao, Yonglun Luo, Chen Li and Subrata Kumar Dey supervised manuscript preparation and edited the manuscript.

## DATA AVAILABILITY STATEMNT

All data used for the analysis in this report are available in the CNGB Nucleotide Sequence Archive (CNSA: https://db.cngb.org/cnsa), Accession Number: CNP0000318.
